The article "Predictive Analysis of Hospital HIS System Usage Satisfaction Based on Machine Learning" was published in 2022. Journal: Comput Math Methods Med.

# Predictive Analysis of Hospital HIS System Usage Satisfaction Based on Machine Learning

**DOI:** 10.1155/2022/1366407

**Published:** 2022-06-14

**Authors:** Yuhang Hu, Haotian Gan

**Affiliations:** ^1^Finance Section, The Second Affiliated Hospital of Qiqihar Medical University, Qiqihar, 161006 Heilongjiang, China; ^2^Computer Centre, The Third Affiliated Hospital of Qiqihar Medical University, Qiqihar, 161006 Heilongjiang, China

## Abstract

Hospital information system (HIS) can provide a full range of information support for various hospital business activities and information collection, processing, and transmission, helping medical service providers. And HIS can reduce medical service costs and improve work efficiency, greatly reducing errors in diagnosis and treatment. Although the advantages of using the HIS are obvious, there are still some challenges in its use, the most prominent being how to make the medical staff use HIS effectively. Based on this background, this paper uses machine learning (ML) technology to predict and analyze the satisfaction of HIS use in hospitals and completes the following work: firstly, introduce the situation and development trend of HIS construction at home and abroad and provide theoretical basis for model design. The related development technologies are discussed and studied in detail. Second, the ML algorithm is used to provide a prediction strategy. The support vector machine (SVM) can handle small data sets well, and this study applies the AdaBoost technique to improve the model's generalization ability and accuracy. Lastly, a diversity metric is included to guarantee that the basic learner has good variety in order to increase the algorithm's performance. Accuracy rates may reach more than 95% in the case of tiny data sets, according to the self-built data set used for testing. This proves the superiority of the model proposed in this paper.

## 1. Introduction

The amount of scientific and technical objects that aid people's lives and work has steadily increased, and informatization has gradually supplanted the intrinsic conventional, with information systems being applied to all aspects of daily life, whether thoroughly or superficially. The deep integration of traditional medical care with information technology and the Internet has generated an entirely new revolution in the medical industry at hospitals, where our health and personal information are firmly linked. Hospitals at all levels have spent a great deal of money in the installation and development of HIS with the full backing of the government. Secondary and tertiary hospitals are now widely accepted, resulting in vastly improved medical care [1].

In 2018, the State Council issued several documents to emphasize the development and improvement of the “Internet+medical and health” service model and to improve the hospital informatization construction and convenience services [2]. HIS can provide comprehensive information support for various hospital operations and information collection, processing, and transmission, and help medical service providers such as doctors, nurses, and hospital management to obtain more timely, accurate, and complete medical information. The reduction of medical service costs and the improvement of work efficiency also greatly reduce the errors of diagnosis and treatment, and ultimately, the improvement of medical quality brings the improvement of patient satisfaction [3]. Despite the apparent benefits of employing the HIS, there are still certain difficulties associated with its implementation. One of the most important is how to make HIS “effectively used” by its direct users, such as physicians, nurses, and hospital managers. Most hospitals these days gauge how well physicians are doing their jobs based on how long they spend treating patients and how accurate their diagnoses are. For the sake of the hospital's efficiency and effectiveness, the HIS should be implemented in order to better support the hospital's entire work flow. However, in their day-to-day duties as doctors, they must also deal with the unique challenges that come with working in a hospital and dealing with a variety of situations that arise due to the unique nature of patient care, including diagnosis, treatment, and follow-up. The standardization of most information systems means that they are not always able to assist medical professionals in dealing with a variety of unique scenarios. Instead, it increases their burden and, in certain cases, decreases their level of agency at work. Since many physicians and other system users, such nurses, simply see the hospital information system as a tool they must use because of the hospital's demands, they are unable to make full use of the system and fail to meet the goals of its deployment [4]. Because of this, it is critical to examine the way in which HIS is used and the impact it has on medical diagnosis and treatment, as well as hospital administration, and to perform an in-depth theoretical exploration of the elements and mechanisms that influence it. Scholars in both the United States and overseas tend to concentrate on how to get people to use information systems from the standpoint of frequency and length of usage, and they tend to focus on enterprise information systems rather than HIS. Studies on information systems' postimplementation stages have become increasingly common in recent years, but there are few studies on the “effective use” of the system in terms of integrating the user's personal characteristics, technical characteristics, and organizational environment in relation to medical scenarios. The research perspective of the “effective use” of the system to explore the influencing factors at different levels is even lacking [5, 6]. Therefore, starting from the special context of the application of information systems to hospitals, this paper explores how personal, technological, and environmental factors affect doctors, nurses, and hospital management based on the classic behavioral theory, technology acceptance model and its extended model. Medical service providers “effectively use” the hospital information system and then combine ML technology to predict and analyze the satisfaction with the use of the HIS, in order to promote the improvement of my country's medical quality and the development of hospital informatization.

The paper organizations are as follows: Section 2 defines the related work.  Section 3 discusses the methods of the proposed concepts.  Section 4 discusses the analysis of experimental results.  Section 5 concludes the article.

## 2. Related Work

The United States is the first country in the world to use the HIS [7]. The United States was the first to introduce computers into hospital management and financial work. After computer engineers continued to improve the software, computers were expanded to all aspects of hospital work and used in various fields of hospitals, such as medical treatment, scientific research, and teaching. And management and other aspects have been comprehensively promoted and finally formed the so-called HIS system. The information system of American hospital is the originator of modern HIS. In the 1990s, the US Department of Defense developed and designed a new generation of HIS system for the US military in hundreds of hospitals and more than 500 clinics around the world [8]. The system can not only share the patient's medical examination results, electronic medical records, and medical imaging data on the Internet, but its biggest feature is that it can realize telemedicine consultation among US military hospitals around the world [9]. HIS research and development in European countries started later but progressed quickly. Almost every European country has succeeded in implementing a standardized HIS, which requires connecting computer terminals across a LAN to build a regional network and then creating an HIS with systematic features. Denmark's “Red System,” for example, and France's “Integrated Hospital Information System” are two of the best examples [10]. A system called “SHINE” is currently being developed by the EU countries represented by Germany, France, the United Kingdom, and Italy, which not only maintains the functional characteristics of the hospital's own information system but also shares information between hospitals in various countries via the Internet [11]. In general, the HIS research in developed countries in Europe and the United States is early and the development speed is fast. It was originally to meet the business needs of the rapid development of the hospital, but in turn, it has promoted the progress of the hospital's work in the continuous practical application.

It is the informatization of hospitals in developed countries, an important part of modernization [12]. The development of hospital informatization can be roughly divided into three stages. The first stage is hospital administrative office management, the second stage is hospital information system, and the third stage is HIS that focuses on medical impact processing, unified medical language system, patient records. HIS is trending towards miniaturization, intelligence, and integration. In the early days of the founding of China, my country's economic foundation and science and technology were relatively backward, and objective factors caused the research on HIS in my country to be nearly 20 years later than that of developed countries in Europe and America. In the 1990s, China began to develop its own HIS. The software enterprise units gradually develop my country's independent HIS system. Although our country started late, the system function basically has the characteristics it should have. Compared with foreign medical standard systems, my country's medical information does not have consistent standards for data information and business processes, which invisibly increases the difficulty and complexity of system development and hinders the sharing of medical information among hospitals [13–15]. Therefore, in the process of building hospital informatization, country should increase capital investment to improve hospital information standardization. This can improve the information interface between the hospital and external institutions and truly realize the integration of hospital information [16, 17]. There are many HIS software development businesses on the market, and the standard specifications and module functionalities of the systems built by different companies are relatively different because there is no unified development standard and specification for the HIS at the moment. In recent years, the HIS has gotten increasingly difficult in order to fulfil modern hospital management, and it is no longer a solution for a single manufacturer. There is an integration problem in the application of products from different manufacturers in the same hospital. And because the functions of the HIS are gradually expanded, different modules use completely different hardware and software technologies, and may be developed by different manufacturers, the management of the entire information system is decentralized, and there is no natural relationship between modules. Moreover, most HIS use the method of parameter definition to solve the problem of software adaptability. Once the parameter definition cannot meet the needs of users, modifying the program may become a catastrophic task [18–21]. In order to meet the needs of parameter definition, the module is very complicated to write, and the modification is prone to new errors. The reason for this confusion is that each HIS development enterprise does not have a unified standard, which makes it difficult to transmit and share information in a “heterogeneous environment.” There is already a mature standard HL7 for text information exchange between HIS in the world. At the same time, there are relatively mature middleware technologies. These standards and technologies are used to build a middle-layer software, which can effectively integrate different information systems and realize the sharing of medical information quickly and easily.

## 3. Method

In this section, we defined the prediction problem analysis and algorithm selection, support vector machines, integrated learning, model creation and algorithm improvement, and hospital HIS use satisfaction index in detail.

### 3.1. Prediction Problem Analysis and Algorithm Selection

#### 3.1.1. Prediction Problem Analysis

The analysis of the satisfaction prediction problem of the HIS in the hospital in this paper is similar to the evaluation problem. The classification process is the prediction process in machine learning. A classification model with machine learning can predict satisfaction. Therefore, using the ML method to predict the satisfaction of hospital HIS use, it is necessary to select an appropriate algorithm and optimize the algorithm. Common ML methods and application scenarios are shown in Figure 1.

The problem of predicting the use satisfaction of hospital HIS is a multiclassification problem, and the classification algorithm in ML can be used. ML includes a variety of classification models and classification algorithms, such as SVM, neural networks, clustering, naive Bayesian algorithms, logistic regression, and decision trees.

#### 3.1.2. Algorithm Selection

By analyzing the commonly used ML classification algorithms and then selecting the appropriate algorithm, the classification algorithm used in this paper should first be a supervised learning algorithm. To evaluate the quality of college students' training in this paper, it is first necessary to preprocess some sample data and analyze the sample data. Labeling is performed and then used for model training. Therefore, several commonly used supervised learning algorithms are compared here. The decision tree algorithm is prone to overfitting, and the accuracy is not high, and the recursive operation of the decision tree takes up a lot of memory. To improve the accuracy of the decision tree by means of ensemble learning, such as using the boosting algorithm, it is necessary to study the depth of the decision tree at this time, and the method is not simple and effective. For logistic regression, the samples need to be linearly separable or nearly linearly separable. When there are many data features, logistic regression is used for classification, and the classification task cannot be better completed due to the low accuracy. Bayesian classification mainly has the following shortcomings. First, because Bayesian classification is based on a probability model, using Bayesian classification requires probability assumptions. If the probability assumptions are not reasonable enough, the final result will be less accurate. At the same time, it is relatively difficult to assume that the probability is relatively difficult, and the data requirements are special. For the same data, if its representation is different, the results will vary greatly. For neural networks, if the amount of data is large, its accuracy is high, but it requires huge data preprocessing work, and if the amount of data is not enough, it will lead to overfitting problems. At the same time, there is no standard for the selection of the number of neurons, and the selection of neurons will have a greater impact on the results. SVM has good generalization ability, is not sensitive to data, and has strong generalization ability on small data and is still applicable to linear inseparable cases, and the modeling is simple and efficient. Therefore, in this paper, support vector machine is selected as the hospital HIS use satisfaction prediction model. Since the accuracy of the SVM still has room for optimization, this paper uses the ensemble learning algorithm AdaBoost to optimize the SVM.

### 3.2. Support Vector Machines

SVMs mainly include support vector classification (SVC) and support vector regression (SVR). The SVC is used for classification problems, while the SVR is mainly used to solve nonlinear regression in regression problems. In this paper, the use satisfaction prediction problem of hospital HIS is essentially a classification problem from the perspective of ML. Therefore, for the ML model of hospital HIS use satisfaction prediction problem, the research should be carried out from the classification model. This paper mainly studies the SVC model.

#### 3.2.1. Algorithm Principle

There are numerous strategies for solving classification problems among supervised learning algorithms. SVMs, for example, have a number of advantages when it comes to tackling classification problems, including high performance on small sample sets and strong generalization capabilities. SVM finds a plane in the sample space, called a hyperplane, so that as many samples belonging to different categories in the sample space can be correctly classified as possible. Finding the hyperplane requires training the model through the training data set and obtaining the hyperplane according to the characteristics of the training data set. After the hyperplane is obtained, it can be used to classify the sample data, and the category to which the test sample belongs is determined according to the position of the sample points in the sample data relative to the hyperplane in space. The sample data in the data set is composed of two parts: feature and category label. In this paper, the feature refers to the hospital HIS use satisfaction index, and the category label refers to the hospital HIS use satisfaction level. It is an ideal state for the hyperplane to perfectly classify the sample points, and many data in reality cannot be perfectly divided into different categories, that is, linear inseparability. In this case we have to allow a small number of points to be misclassified. According to the actual situation of the problem, “slack variables” are introduced to allow some sample points to be misclassified within an acceptable range. Searching for a hyperplane during training allows a small number of points that cannot be fully classified, so it is necessary to find the best possible hyperplane. In reality, data is a variety of data forms and dimensions and also has its own characteristics. Some data sets are inseparable in their original dimensions. For indivisible data, it is usually to find a higher dimension so that the sample points can be mapped from the original dimension to higher dimensions so that the samples are separable. The algorithm grows more difficult as the number of dimensions increases, occasionally leading to insurmountable issues. At this point, we must apply the kernel function to map low-dimensional data to high-dimensional space in order to separate the data points in the high-dimensional space and avoid the problem of increasing the difficulty of calculation in the high-dimensional space. The selection of kernel function is very important for the performance of SVM. Inappropriate selection of kernel function will lead to poor final classification effect.

Let the hyperplane *w*^*T*^*x* + *b* = 0 in the space, where *w* the normal is vector and *b* is the displacement term. When the samples are linearly separable, there may be more than one hyperplane that can correctly classify the samples.

There are multiple hyperplanes that can correctly distinguish samples, and the hyperplane is the farthest from the points in the sample, which we call the optimal hyperplane. Let the distance from the sample to the optimal hyperplane be *d*, and the distance formula from the sample point to the optimal hyperplane can be obtained from the formula of the distance from the point to the plane as follows.

(1) $$\begin{array}{c} d=\frac{\left|w^{T}x+b\right|}{\left\|w\right\|}. \end{array}$$

Let *D* be the training sample set, *D* = {(*x*_*i*_, *y*_*i*_)|*i* = 1, 2, 3, ⋯, *n*}, where *x*_*i*_ ∈ *R*^*d*_0_^, *y*_*i*_ ∈ {−1, 1}, *d*_0_ is the input sample dimension, this paper refers to a scalar number, and *n* is the number of samples. If the hyperplane can correctly classify the samples, *w*^*T*^*x* + *b* > 0 can be obtained for the positive example, i.e., *y*_*i*_ = +1, and *w*^*T*^*x* + *b* < 0 for the negative example. Therefore, for the positive and negative examples, the following formula can be obtained.

(2) $$\begin{array}{c} \left\{\begin{array}{cc} w^{T}x_{i}+b\geq +1, & y_{i}=+1,\\ w^{T}x_{i}+b\leq -1, & y_{i}=-1. \end{array}\right. \end{array}$$

In a schematic diagram of SVM with interval and hyperplane, there will be a point that is closest to the solid line in the hyperplane graph, and these sample points make the equal sign in formula (2) true. Such a sample point is called a support vector, and the distance and interval from the support vector to the hyperplane are represented by *F*, which can be calculated by

(3) $$\begin{array}{c} F=\frac{2}{\left\|w\right\|}, \end{array}$$

when *F* achieves the maximum value, the support vector of the positive example and the support vector of the negative example are the farthest from the hyperplane, and the hyperplane can better classify the samples. Therefore, the search for the optimal hyperplane is converted into the value of *w* and *b* when the value of *F* is maximized. In order to facilitate the calculation, it is converted into the following

(4) $$\begin{array}{c} \underset{w,b}{\min}\frac{1}{2}{\left\|w\right\|}^{2},s.t.y_{i}\left(w^{T}x_{i}+b\right)\geq 1,i=1,2,\cdots ,n. \end{array}$$

The hyperplane can be obtained by solving the formula (4), and the classification of the samples can be realized according to the obtained hyperplane formula as a SVM model. Solving formula (4) usually uses the Lagrange multiplier method. Therefore, the first task of the SVM classification model is to use the training set data to determine the hyperplane and obtain the hyperplane formula. SVM can be simply understood as a mapping relationship from sample features to classification results. In this paper, it is a mapping relationship from the satisfaction prediction data used by the hospital HIS to the prediction results. SVM training refers to finding the connection between data features and classification outcomes by solving this mapping relationship using processed sample data. This paper uses Figure 2 to describe the process of SVM to solve hyperplane.

The solution of formula (4) is actually the solution of a quadratic programming problem, and its dual problem is obtained by using the Lagrange multiplier method, and the solution is solved by combining the KKT conditions. Using the Lagrange multiplier method to solve formula (4), the Lagrange function can be obtained as

(5) $$\begin{array}{c} L\left(w,b,\lambda \right)=\frac{1}{2}{\left\|w\right\|}^{2}+\overset{n}{\underset{i=1}{\sum }}\lambda_{i}\left(1-y_{i}\left(w^{T}x+b\right)\right). \end{array}$$

Solving the partial derivatives of formula (5) yields

(6) $$\begin{array}{c} \frac{\partial L\left(w,b,\lambda \right)}{\partial w}=w-\overset{n}{\underset{i=1}{\sum }}\lambda_{i}y_{i}x_{i}, \end{array}$$

(7) $$\begin{array}{c} \frac{\partial L\left(w,b,\lambda \right)}{\partial b}=\overset{n}{\underset{i=1}{\sum }}\lambda_{i}y_{i}. \end{array}$$

By making formulas (6) and (7) zero, formulas (8) and (9) can be obtained as follows.

(8) $$\begin{array}{c} w=\overset{n}{\underset{i=1}{\sum }}\lambda_{i}y_{i}x_{i}, \end{array}$$

(9) $$\begin{array}{c} 0=\overset{n}{\underset{i=1}{\sum }}\lambda_{i}y_{i}. \end{array}$$

Simultaneous formulas (8) and (5), eliminating *w* and *b* in formula (5), the dual problem of formula (4) can be obtained

(10) $$\begin{array}{c} \underset{\lambda }{\max}\overset{n}{\underset{i=1}{\sum }}\lambda_{i}-\frac{1}{2}\overset{n}{\underset{i=1}{\sum }}\overset{n}{\underset{j=1}{\sum }}\lambda_{i}\lambda_{j}y_{i}y_{j}x_{i}^{T}x_{j},s.t.0=\overset{n}{\underset{i=1}{\sum }}\lambda_{i}y_{i}. \end{array}$$

The solution of formula (10) satisfies the KKT condition, and the analysis shows that only the *λ*_*i*_ value corresponding to the support vector (*x*_*i*_, *y*_*i*_) is not 0, and the rest *λ*_*i*_ values are 0. After solving *λ*_*i*_^∗^, the optimal *w*^∗^ and *b* are obtained

(11) $$\begin{array}{c} w^{*}=\overset{n}{\underset{i=1}{\sum }}\lambda_{i}^{*}y_{i}x_{i}, \end{array}$$

(12) $$\begin{array}{c} b=1-w^{*T}x. \end{array}$$

The hyperplane formula can be obtained. For cases that are close to linearly separable or linearly inseparable in low dimensions, slack variables and kernel functions are introduced. There are many choices of kernel functions, and different kernel functions can be selected according to specific problems, or a new kernel function can be constructed. In the same way as the above solution method, after introducing the slack variable and the kernel function, the optimal classifier can be obtained by the Lagrange multiplier method, as shown in the following formula.

(13) $$\begin{array}{c} f\left(x\right)=\overset{n}{\underset{i=1}{\sum }}\lambda_{i}^{*}y_{i}K\left(x_{i},x\right)+b^{*}. \end{array}$$

#### 3.2.2. Support Vector Machine Multiclassification

The SVM is a binary classifier, as shown by the analysis of the SVC principle, and the hospital HIS use satisfaction prediction problem in this paper is a multiclassification problem. In order to apply the SVM to the multiclassification problem, it is necessary to use SVMs to construct multiple classifiers. The usual methods include the direct method and the indirect method. Due to the high computational complexity of the direct method and the difficulty in implementation, the direct method is generally not used, and the indirect method is usually used to construct multiple classifiers. The indirect method has the following two strategies.

*(1) Indirect Multiclassification Strategy*. For other one-versus-rest (OVR) training samples, construct multiple SVMs to take a certain category as one class and train the other classes as one class, so that *m* categories are constructed by constructing *m* support vector machines. When classifying the samples, different SVMs on the sample classification decision function value classify the unknown samples into the class with the largest classification function value. The samples are separated into four groups in the hospital HIS use satisfaction prediction; therefore, the SVM is used for four categories of classification and a pair of additional classification algorithms are applied.  Figure 3 is shown below. The four SVMs are SVM-1, SVM-2, SVM-3, and SVM-4, respectively, and the corresponding four categories are A, B, C, and D.

For a pair of other classification strategies, when classifying each class, there will be fewer positive samples than negative samples. When there are a lot of classes, the number of positive and negative samples in each binary classifier is asymmetric, which leads to classification and recognition. The difficulty increases, and the final output result is to make a decision by comparing the output results of several classifiers and selecting the maximum value. The output results of the same classifier are comparable, but the output results of different classifiers are not comparable, thus leading to wrong decisions.

*(2) Indirect Multiclassification Strategy*. For one-versus-one (OVO), the OVO classification method constructs an SVM classifier between any two categories, so that for multiclassification problems with*m*categories, in total,*m*(*m* − 1)/2classifiers need to be constructed. When an unknown category is input, *m*(*m* − 1)/2 classifiers vote according to their respective classification results, and the final result is the category with the most votes. Taking the four classifications in this article as an example, the schematic diagram of the OVO classification method is shown in Figure 4.

This method is widely used and has high classification accuracy. However, due to the large number of classifiers constructed, the cost is also high. However, when the experimental conditions permit, this method can obtain higher accuracy. The categorization in this study will be done using the OVO approach, which has a high level of accuracy. And, compared to a pair of other approaches, there are only two extra classifiers because there are only four classification results. The computational cost is acceptable, and the classification accuracy should be improved as much as possible.

### 3.3. Integrated Learning

#### 3.3.1. Principle of Ensemble Learning

Ensemble learning, in simple terms, is to combine multiple learners to improve the overall performance of multiple learning models. As a hotspot of ML, ensemble learning is listed by authoritative scholars as the first of the four research directions in the field of ML. Using the ensemble learning algorithm to integrate and combine simple learners, the learning effect and performance are improved. According to the different combination methods, ensemble learning can be divided into two categories: “homogeneous” and “heterogeneous.” The learners in the homogeneous ensemble method are of the same type, and the learners in the heterogeneous ensemble method are of different types, and the learners in the homogeneous ensemble method can also be called basic learners. The learners in heterogeneous ensembles are called “component learners” or individual learners.

#### 3.3.2. Ensemble Learning Category

Homogeneous type of ensemble learning is usually used for different training sets or random sampling of the original data set, so that the training set on each individual learner is different. According to the techniques used by homogeneous types of individual learners to obtain different training samples, they can be divided into methods such as resampling the training set, manipulating input variables, and manipulating output targets. There are two generation methods for individual learners. If there is a strong dependency between individual learners, the generation method is serial. If there is no strong dependency, the individual learners can be generated in parallel. The former is represented by boosting, and the latter is represented by bagging and “random forest.”

#### 3.3.3. AdaBoost Algorithm

With its solid theoretical foundation, high accuracy, and simplicity, AdaBoost, the most recognized algorithm in ensemble learning, has been widely applied in various domains and has achieved significant success. AdaBoost primarily uses numerous iterations to create an ensemble learning model. It can adjust the component learner in an adaptive way, and the AdaBoost algorithm updates the weight of the sample of each iteration.

### 3.4. Model Creation and Algorithm Improvement

There is currently no fixed method for the selection of the kernel function, which is usually selected based on experience and comparison. According to general experience, the selection of the kernel function usually first selects the linear kernel function, and if the effect is not ideal, the Gaussian kernel function can be used. The SVM kernel function that is not used for integration in this paper selects the linear kernel function for better classification. The linear kernel function is *k*, and the constant *C* and *C* ≥ 0 are introduced in the way of “soft interval,” and the slack variable *r* ≥ 0 is introduced. Through the method mentioned above, the final decision formula can be obtained as shown in formula (14), and the coefficients in the formula can be obtained by the data operation in the training set.

(14) $$\begin{array}{c} f\left(x\right)=\overset{n}{\underset{i=1}{\sum }}\lambda_{i}^{*}y_{i}K\left(x_{i},x\right)+b^{*},w^{*}=\overset{n}{\underset{i=1}{\sum }}\lambda_{i}^{*}y_{i}x_{i},b^{*}=1-w^{*T}x \end{array}$$

Part of the sample data is used as the test data, and the student's index value is input into formula (14) to output the final discrimination result. In this paper, the OVO strategy is used to achieve multiclassification, and the accuracy of the model is measured by comparing the output results with the actual category of the sample.

This section studies the integration of the AdaBoost algorithm and the SVM algorithm. By selecting the kernel function of the SVM and setting its parameters, the accuracy is reduced and the characteristics of the boosting algorithm are satisfied, thereby improving the performance of the integrated model. And the diversity measurement of the SVM algorithm makes it have better diversity and further improves the efficiency and performance of the integrated algorithm.

#### 3.4.1. Based on the Diversity of Learning Algorithms

As the most famous algorithm in the boosting algorithm, AdaBoost has some characteristics of the boosting algorithm. The boosting algorithm requires the basic learners to have the characteristics of diversity. Only when the basic learners have good diversity can the ensemble learning model have better classification results. Therefore, its diversity is guaranteed, that is, the basic learners are not correlated, so that the performance of the final ensemble model can be optimized. Scholars have studied the diversity of base learners from different perspectives. The first is how to define the diversity of classifiers, what diversity is, how to measure it, and what conditions are met to be diverse. The second is how to introduce a diversity measure when creating an ensemble learning model to create a multiclassifier system. Finally, it is studied under which conditions the diversity of base classifiers achieves the optimal performance of the ensemble model. For the diversity of the ensemble learning AdaBoost-SVM base learner, we define it as follows. For the *t*th component classifier, the diversity *d*_*t*_ on the sample *X*_*i*_ is calculated by

(15) $$\begin{array}{c} d_{t}=\begin{array}{cc} 0, & \text{if }h_{t}\left(X_{i}\right)=f\left(X_{i}\right),\\ 1, & \text{if }h_{t}\left(X_{i}\right)\neq f\left(X_{i}\right), \end{array} \end{array}$$

where *h*_*t*_(*X*_*i*_) is the output result of the *t*th classifier on sample *X*_*i*_, and *f*(*X*_*i*_) is the label of sample *X*_*i*_. The diversity *D*_*iv*_ of the *T* component classifiers of AdaBoost-SVM on *N* samples can be calculated by

(16) $$\begin{array}{c} D_{iv}=\frac{1}{TN}\overset{T}{\underset{t=1}{\sum }}\overset{N}{\underset{i=1}{\sum }}d_{t}\left(X_{i}\right). \end{array}$$

#### 3.4.2. Kernel Function and Parameters

Boosting algorithm, as the learning algorithm of its basic learner, has poor classification performance, and the accuracy of classification is better than that of random guessing, that is to say, it requires a basic learner. The accuracy is just above 0.5. In general, SVM has a better classification effect. In this way, the integration of SVM algorithm with AdaBoost algorithm seems to be contrary to the principle of boosting. Therefore, if SVM is used as the base learner of the AdaBoost algorithm, then there must be a way to reduce the accuracy of SVM and be above 0.5. The research on the SVM algorithm shows that the accuracy of the SVM algorithm is affected by the selected kernel function and parameters. In the SVM that selects the Gaussian kernel function, the classification performance is affected by the regularization parameter *C* and the Gaussian bandwidth *W*. When the value of *C* is small, the performance of the algorithm is greatly affected by *W*. Therefore, when the value of *C* is roughly suitable, the performance of the algorithm can be more effectively changed by the value of parameter *W*. When the value of *W* is relatively large, the classification performance of SVM will be appropriately weakened. Therefore, at the beginning of the iteration of the AdaBoost algorithm, an appropriately large value of *W* should be given, and the value of *W* should be modified after each iteration.

#### 3.4.3. AdaBoost-SVM Algorithm

We optimize AdaBoost-SVM through diversity and accuracy of base learners. For the diversity of each base learner, we will get a value *D*_iv_ that measures the diversity; it can be seen in the above algorithm that a threshold DIV is set for diversity. If *D*_iv_ is greater than the threshold DIV set above, the current base learner can be added to the ensemble learning model as a new learner. Otherwise, the current base learner needs to be discarded. Compared with the original AdaBoost algorithm, the base learner has better diversity to build an ensemble learning model, and the generalization ability and efficiency of the final ensemble model will be improved.

### 3.5. Hospital HIS Use Satisfaction Index

For the prediction of hospital HIS usage satisfaction proposed by the subject of this paper, it is necessary to construct a quantifiable evaluation index. By referring to the relevant literature and combining with the development status of the hospital HIS, the constructed evaluation indicators are shown in Table 1.

## 4. Experiment and Analysis

In this section, we defined the data set and model training and experimental accuracy of different models in detailed.

### 4.1. Data set and Model Training

To verify the effectiveness of satisfaction prediction model proposed in this paper, this paper builds a dataset. This dataset contains 900 sets of data. This work uses Python and scikit-learn framework to construct a network. When the SVM selects the Gaussian kernel function, *W* = 35, *C* = 1.4, and the number of basic learners is 8, the error rate of the model output reaches the lowest, and the final error rate output of the AdaBoost-SVM model is 0.05, that is, the accuracy rate is 0.95. The training results of the AdaBoost-SVM model are shown in Figure 5.

As can be observed from running data, the model's error rate on the test and training sets does not change whether there are 8 component learners in the model. In other words, after the 8 basic learners are built, the model's error rate approaches the ideal level under the specified parameters. The model's test set error rate is 0.05 when the curves are balanced. The curve does not alter after increasing the number of base classifiers. As a result, there are eight primary classifiers. HIS-based AdaBoost-SVM assessment model is assessed using the data from the satisfaction data sample, except for training and test samples, with four sets of 30 samples each.  Table 2 shows the test findings.

Table 2 shows the sample data for four categories, with 30 samples for each category to evaluate the model. After entering the model, for A-level satisfaction, the number of correct classifications is 26, and the number of wrong classifications is 4, of which 1 is wrongly classified into category B and 2 samples are wrongly classified into category C. In satisfaction level B, 29 samples were correctly classified and one sample was wrongly classified into class C. For C-level satisfaction, 28 samples were correctly classified, and the remaining two samples were wrongly classified into B and D categories, respectively. For D-level satisfaction, the number of correctly classified samples is 28 and the number of misclassified samples is 2 and misclassified into class A. It can be concluded that the AdaBoost-SVM evaluation model has good performance in both accuracy and recall. After training, the model can be easily used to predict the satisfaction of HIS usage.

### 4.2. Experimental Accuracy of Different Models

We use Python language to test the SVM, AdaBoost-SVM, and BP neural network with the help of scikit-learn ML framework. The test data set still uses the data set built in this paper. There are 900 data samples in this data set, each sample has 4 features, and the samples have three categories in total. By testing the algorithm, the relationship between the accuracy of the algorithm and the number of samples can be obtained as shown in Figure 6. In the experiment, the parameter selection *C* of SVM is 10, the kernel function selects the Gaussian kernel function parameter *W* = 14, and the parameters in AdaBoost-SVM select *C* = 10, *W* = 14, and DIV = 0.3. The activation function of the BP neural network uses the Relu activation function, and the threshold *T* = 0.005.

It can be seen from the test results that the accuracy rate of AdaBoost-SVM is the highest, and can reach more than 95%, and the accuracy rate of SVM is higher than that of BP neural network. Therefore, the AdaBoost-SVM algorithm is selected in this paper, which can reduce a lot of data preprocessing work and make the accuracy of the model to be optimal in the case of a small amount of data. It can effectively avoid heavy data processing work due to the need for a large number of data samples for model training in the prediction of hospital HIS use satisfaction.

## 5. Conclusion

The information era has arrived in the twenty-first century, and the HIS is a medical service-oriented information system that is part of this trend. Aside from some important manual procedures, most hospitals have essentially completed the transition from traditional management to computerized automatic management, which decreases medical staff workload and enhances labor efficiency and service quality. Accurate and standardized computerized management provides scientific data prediction and information decision-making for the medical industry. HIS usage as a research context and the idea of user pleasure as a research object are examined in this study. Based on the technology acceptance model and rational and planned behavior theory, this research investigates the characteristics of the human, technical, and organizational environment that determine the successful use of HIS. In this paper, the current popular ML method is used to predict the current use satisfaction of HIS through the constructed HIS use satisfaction evaluation index. The work done in this thesis includes the following aspects: (1) introduce the current state of HIS construction at home and overseas, as well as the challenges that exist in our country's HIS, and make some recommendations. To prepare for the upcoming model design, the theoretical foundation and related development technologies required for model design are addressed and examined in depth; (2) analyze the prediction method and introduce the algorithm of machine learning as the prediction method. This work uses the AdaBoost method to select and integrate SVMs to increase accuracy and generalization even further since SVMs do well on small data sets and still have potential for improvement. This study picks the Gaussian kernel function and modifies the SVM parameters such that the SVM's accuracy may match the criteria of the AdaBoost method when it is employed as the base learner of the AdaBoost algorithm; and (3) a diversity metric is introduced to ensure that the basic learner has good diversity in order to increase the algorithm's performance. The accuracy rate of AdaBoost-SVM can reach more than 95% in the event of a little amount of data, according to the self-built data set used to test the algorithm. This demonstrates the model provided in this paper's superiority.

## Figures and Tables

**Figure 1:** Application scenario of machine learning algorithms.

**Figure 2:** Support vector machine to solve the hyperplane flow chart.

**Figure 3:** Schematic diagram of OVR strategy.

**Figure 4:** Schematic diagram of OVO classification method.

**Figure 5:** The training results of the AdaBoost-SVM model.

**Figure 6:** Experimental accuracy of different models.

**Table 1:** Satisfaction index of hospital HIS system use.

First-level indicator	Secondary indicator	Label
System security	Use database super user login method	X1
	Program provides data backup function	X2
	Provide full monitoring of data modification	X3
System scalability	Provide various parameters to fully adjust system	X4
	Subsystems can operate individually or shared	X5
	Provide various external interfaces	X6
System maintainability	Easy and fast system installation	X7
	Provides tools for maintaining databases	X8
	Client and system automatic upgrade	X9
Software ease of use	Has a unified operation interface	X10
	With personalization function	X11
	Provide online help	X12
External interface	Statistics related system interface	X13
	With medical insurance interface	X14
	Disease control and health monitoring interface	X15

**Table 2:** Sample classification situation.

Satisfaction level	Number of samples	Evaluation results			
		A	B	C	D
A	30	26	01	02	01
B	30	0	29	01	01
C	30	0	01	28	01
D	30	02	0	0	28

## Data Availability

The data sets used during the current study are available from the corresponding author on reasonable request.
